RETRACTED

# The Significance of Notch1 Compared with Notch3 in High Metastasis and Poor Overall Survival in Hepatocellular Carcinoma

**DOI:** 10.1371/journal.pone.0057382

**Published:** 2013-02-28

**Authors:** Liang Zhou, Ning Zhang, Wenjie Song, Nan You, Qingjun Li, Wei Sun, Yong Zhang, Desheng Wang, Kefeng Dou

**Affiliations:** Department of Hepatobiliary Surgery, Xijing Hospital, The Fourth Military Medical University, Xi’an, Shannxi, People’s Republic of China; The University of Hong Kong, Hong Kong

## Abstract

**Background:**

The prognosis for patients with hepatocellular carcinoma (HCC) is poor, and the mechanisms underlying the development of HCC remain unclear. Notch1 and Notch3 may be involved in malignant transformation, although their roles remain unknown.

**Materials and Methods:**

HCC tissues were stained with anti-Notch1 or -Notch3 antibody. The migration and invasion capacities of the cells were measured with transwell cell culture chambers. RT-PCR was used to measure the expression of Notch1 and Notch3 mRNA. Additionally, western blot analysis was used to assess the protein expression of Notch1, Notch3, CD44v6, E-cadherin, matrix metalloproteinase-2 (MMP-2), MMP-9, and urokinase-type plasminogen activator (uPA). RNA interference was used to down-regulate the expression of Notch1 and Notch3. Cell viability was assessed using MTT.

**Results:**

Based on immunohistochemistry, high Notch1 expression was correlated with tumor size, tumor grade, metastasis, venous invasion and AJCC TNM stage. High Notch3 expression was only strongly correlated with metastasis, venous invasion and satellite lesions. Kaplan-Meier curves demonstrated that patients with high Notch1 or Notch3 expression were at a significantly increased risk for shortened survival time. In vitro, the down-regulation of Notch1 decreased the migration and invasion capacities of HCC cells by regulating CD44v6, E-cadherin, MMP-2, MMP-9, and uPA via the COX-2 and ERK1/2 pathways. Down-regulation of Notch3 only decreased the invasion capacity of HCC cells by regulating MMP-2 and MMP-9 via the ERK1/2 pathway.

**Conclusions:**

Based on the migration and invasion of HCC, we hypothesize that targeting Notch1 may be more useful than Notch3 for designing novel preventive and therapeutic strategies for HCC in the near future.

## Introduction

Currently, systemic chemotherapy is ineffective in hepatocellular carcinoma (HCC), as evidenced by low response rates and no demonstrated survival benefit. Additionally, liver transplantation is considered the only curative treatment option for HCC. However, its use has been restricted by factors such as the scarcity of donor organs and the risks associated with primary hepatic resection. Many patients undergo different therapies, yet the prognosis of HCC remains dismal, which is mainly attributed to the aggressive metastasis and recurrence of HCC [1]. However, the mechanisms underlying the development of HCC remain unclear.

RETRACTED

The Notch pathway is important for cell fate determination, tissue patterning and morphogenesis, and cell differentiation, proliferation and death [2]. Most studies have focused on Notch1 and Notch3, which may be involved in malignant transformation. Notch1 has been shown to be up-regulated in prostate cancer, small cell lung cancer, pancreatic cancer and HCC and is involved in tumor cell invasion in pancreatic cancer, lingual squamous cell carcinoma, and breast cancer [3]–[8]. Additionally, high Notch1 expression has been reported to be related to poor overall survival rates in breast and colorectal cancer [9], [10]. Aberrant Notch3 expression has been reported in virtually all cases of T cell acute lymphoblastic leukemia (T-ALL), colorectal cancer, HCC, lung cancer, pancreatic cancer, and ovarian cancer [11]–[16]. However, the relationship among Notch1 or Notch3, clinicopathological manifestations and the survival rate in patients with HCC has not been explored. Furthermore, the potential mechanisms of Notch1 and Notch3 involvement in HCC are unclear.

In the present study, we investigated Notch1 and Notch3 expression in HCC tissues and, for the first time, explored the possible relationships between Notch1 and Notch3 expression and prognosis in HCC. We further explored the potential mechanism of Notch1 and Notch3 involvement in the migration and invasion of HCC in vitro.

## Materials and Methods

### Patients and Tissue Specimens

Tissue specimens from HCC and adjacent non-cancerous hepatic tissues (at least 1.5 cm away from the tumor) were collected from 86 patients who underwent surgical treatment for primary HCC in the Department of Hepatobiliary Surgery at Xijing Hospital (Xi’an, China) between 2004 and 2007. Specimens were collected from patients who had not received preoperative treatment. There were 54 male and 32 female patients, with a median age of 45.3 years (range, 30–80 years). This study was approved by the Ethics Committee of the Fourth Military Medical University and conformed to the ethical guidelines of the 2004 Declaration of Helsinki. Written informed consent was obtained from each patient or his or her legal guardians. Clinical parameters, such as gender, age, tumor location, tumor size, tumor grade, metastasis, satellite lesions, tumor number, AJCC TNM stage, and AFP, were collected. In patients diagnosed with metastasis, we also analyzed vascular invasion. Among the 24 cases diagnosed with metastasis, complications included venous invasion (n = 16), bile duct tumor thrombi (n = 9) and lymph node metastasis verified by pathological analysis (n = 4). Enrolled patients were followed for 5 years for survival calculations.

RETRACTED

### Cell Culture and Reagents

A human liver non-tumor cell line (HL-7702, obtained from the Cell Bank of Type Culture Collection of Chinese Academy of Sciences) and HCC cell lines (HepG2, and SMMC-7721, obtained from the Cell Bank of Type Culture Collection of Chinese Academy of Sciences and MHCC97H, obtained from the Liver Cancer Institute of Fudan University) were cultivated in DMEM supplemented with 10% fetal calf serum (Sigma Chemical Co., St. Louis, MO). The cells (1 × 105 cells/well) were seeded into 6-well cell culture plates for 48 h until the next experiments. Primary antibodies against Notch1, Notch3, E-cadherin, matrix metalloproteinase-2 (MMP-2), MMP-9, urokinase-type plasminogen activator (uPA), cyclooxygenase-2 (COX-2) and GAPDH were purchased from Santa Cruz Biotechnology (Santa Cruz, CA, USA). Primary antibodies against CD44v6, extracellular signal-regulated kinase 1 and 2 (ERK1/2) and p-ERK1/2 were purchased from Abcam (Cambridge, UK). All secondary antibodies were obtained from Pierce (Rockford, IL, USA). An SP immunostaining kit purchased from ZYMED (ZSGB; Beijing, China) was used. Notch1 small interfering RNA (siRNA), Notch3 siRNA and an siRNA control were obtained from Santa Cruz Biotechnology (Santa Cruz, CA, USA). To inhibit endogenous COX-2 activity, 50 µmol/l NS-398 (Sigma-Aldrich) and 70 nmol/l SC58125 (Ann Arbor, MI) were used. To inhibit ERK1/2 activity, 10 µmol/l PD98059 (Calbiochem, San Diego, CA) and 1 µmol/l U0126 (Ellisville, Missouri, USA) were used. NS-398, SC-58125, PD98059, and U0126 were dissolved in DMSO (Sigma-Aldrich). All other chemicals and solutions were purchased from Sigma-Aldrich, unless otherwise indicated.

### Immunohistochemistry and Evaluation of Staining

Immunohistochemistry involved the use of the avidin-biotin-peroxidase complex method on all tissues. All sections were deparaffinized in xylene and dehydrated through a graduated alcohol series before endogenous peroxidase activity was blocked with 0.5% H_2_O_2_ in methanol for 10 min. Nonspecific binding was blocked by incubating sections with 10% normal goat serum in PBS for 1 h at room temperature. Without washing, sections were incubated with anti-Notch1 or anti-Notch3 (1∶50) in PBS at 4°C overnight in a moist box. The sections were incubated with biotinylated IgG for 2 h at room temperature and detected with a streptavidin-peroxidase complex. The brown color indicative of peroxidase activity was obtained by incubating the section with 0.1% 3,3-diaminobenzidine in PBS with 0.03% H_2_O_2_ for 10 min at room temperature. The tissue specimens were scored independently by two pathologists blinded to the clinicopathology and outcome of the patients using an immunoreactivity score system described previously [10]. Based on the score, we divided all HCC specimens into two subgroups: the low expression group (score of 0–4) and the high expression group (score of 5–12 score).

RETRACTED

### Small Interfering RNA Transfection

According to the LipofectAMINE 2000 protocol (Carlsbad, CA, USA), HCC cells were transfected with Notch1 siRNA, Notch3 siRNA or control siRNA. The cells transfected with siRNA (1 × 105 cells/well) were seeded into 6-well cell culture plates and allowed to continue growing for 24 h before harvesting for further analysis.

### Real-time Reverse Transcription PCR

Total RNA was extracted and reverse transcribed. The primers used in the PCR are as follows: Notch1, forward primer (5′-CACCCATGACCACTACCCAGTT-3′) and reverse primer (5′-CCTCGGACCAATCAGAGATGTT-3′); Notch3, forward primer (5′-AAGGACGTGGCCTCTGGT-3′) and reverse primer (5′-TCAGGCTCTCACCCTTGG-3′); GAPDH, forward primer (5′- AAATCCCATCACCATCTTCC-3′) and reverse primer (5′- TCACACCCATGACGAACA-3′). The primers were evaluated by running a virtual PCR, and the primer concentration was optimized to avoid primer dimer formation. Additionally, dissociation curves were evaluated to avoid nonspecific amplification. Real-time PCR amplifications were undertaken in the Mx4000 Multiplex QPCR System (Stratagene, La Jolla, CA) using 2×SYBR Green PCR Master Mix (Applied Biosystems). Data were analyzed according to the comparative *C*_t_ method and normalized by the GAPDH expression in each sample.

### Protein Extraction and Western Blotting

The cells were lysed in lysis buffer [8] after incubation for 20 minutes at 4°C. The protein concentration was determined using the Bio-Rad assay system (Bio-Rad, Hercules, CA, USA). Total proteins were fractionated using SDS-PAGE and transferred onto nitrocellulose membrane. The membranes were blocked with 5% nonfat dried milk or bovine serum albumin in 1×TBS buffer containing 0.1% Tween 20 and then incubated with appropriate primary antibodies. Horseradish peroxidase–conjugated anti-rabbit or anti-mouse IgG was used as the secondary antibody, and the protein bands were detected using the enhanced chemiluminescence detection system (Amersham Pharmacia Biotech). The quantification of western blots was performed using laser densitometry, and relative protein expression was normalized to GAPDH levels.

### MTT Assay

The treated cells (1×10^4^ cells/well) were seeded into 96-well cell culture plates and grown for up to 48 h. Cell viability was assessed using the 3-(4,5-dimethyl-2-thiazolyl)-2,5-diphenyl-2H-tetrazolium bromide (MTT) assay (Sigma Chemicals Co.) in accordance with the manufacturer’s protocol. Each experiment included six replications and was repeated three times. The data were summarized as means ± SDs.

RETRACTED

### Migration and Invasion Assays

Cell migration and invasion were analyzed using non-matrigel-coated or matrigel-coated transwell cell culture chambers (8 µm pore size) (Millipore, Billerica, MA, USA). Briefly, treated cells (5 × 10^4^ cells/well) were serum starved for 24 h and plated in the upper insert of a 24-well chamber in serum-free medium. Medium containing 10% serum as a chemoattractant was added to the well, and the cells were incubated for 24 h. Cells on the upper side of the filters were mechanically removed by scrubbing with a cotton swab. The membrane was subsequently fixed with 4% formaldehyde for 10 min at room temperature and stained with 0.5% crystal violet for 10 min. Finally, invasive and migrated cells were counted at 200× magnification in 10 different fields of each filter.

### Statistical Analysis

Statistical analysis was conducted using SPSS 15.0 software (Chicago, IL, USA). Each experiment was repeated at least three times. All data were summarized and presented as means ± SDs. The differences among means were analyzed statistically using a t-test. Associations between Notch1 and Notch3 expression and categorical variables were analyzed using χ^2^ tests and Fisher’s exact tests, as appropriate. Survival curves were calculated using the Kaplan-Meier method and compared using the log-rank test. The Cox proportional hazard model was used for univariate and multivariate analysis to explore the effect of clinicopathological factors and Notch1 and Notch3 expression on survival. P<0.05 was considered statistically significant.

## Results

### Notch1 and Notch3 Immunohistochemistry

Notch1 and Notch3 were mainly localized in the cytoplasm and cell membrane. Neither Notch1 nor Notch3 was significantly expressed in adjacent non-cancerous hepatic tissues, with only weak staining of Notch1 and Notch3 in the cell membrane and cytoplasm. As Fig. 1 (a–h) shows, the expression of Notch1 and Notch3 was different in HCC tissues. Notch1 staining was not detected in 9 samples of HCC. In contrast, weak positive staining of Notch1 was detected in 31 samples of HCC, moderate positive staining was detected in 17 samples, and strong positive staining was detected in 29 samples. Notch3 staining was not detected in 11 samples of HCC. In contrast, weak positive staining of Notch3 was detected in 30 samples of HCC, moderate positive staining was detected in 19 samples, and strong positive staining was detected in 26 samples.

RETRACTED

**Figure 1:** Expression of Notch1 and Notch3 in HCC tissues and Kaplan-Meier statistical analyses of postoperative survival curves according to Notch1 and Notch3 expression. Notch1 expression in HCC tissues (a–d): (a) negative, (b) weakly positive, (b) moderately positive, (d) strongly positive. Notch3 expression in HCC tissues (e-h): (e) negative, (f) weakly positive, (g) moderately positive, (h) strongly positive. (i) Kaplan-Meier statistical analyses of postoperative survival curves according to Notch1 expression; (j) Kaplan-Meier statistical analyses of postoperative survival curves according to Notch3 expression.

### Relationship between Notch1 and Notch3 Expression and Clinicopathological Characteristics

We divided the 86 patients into two subgroups: a high Notch1 or Notch3 expression group and a low Notch1 or Notch3 expression group. The relationship between Notch1 and Notch3 expression and clinicopathological factors is summarized in Table 1. The results showed that high Notch1 expression was strongly correlated with tumor size (P<0.001), tumor grade (P = 0.003), metastasis (P = 0.045), venous invasion (P = 0.014) and AJCC TNM stage (P<0.001). However, the high expression of Notch3 was only strongly correlated with metastasis (P = 0.002), venous invasion (P = 0.010) and satellite lesions (P = 0.033).

**Table 1:** Association of Notch1 or Notch3 expression with clinicopathologic factors of the HCC patients.

Tumor characteristic	n	Notch1		p-value	χ^2^	Notch3		p-value	χ^2^
		High(5–12 score)	Low(0–4 score)			High(5–12 score)	Low(0–4 score)		
All cases	86	46(53.5%)	40(46.5%)			45(52.3%)	41(47.7%)		
Gender									
Male	54	29(53.7%)	25(46.3%)	0.959	0.003	27(50.0%)	27(50.0%)	0.575	0.315
Female	32	17(53.1%)	15(46.9%)			18(56.3%)	14(43.8%)		
Age (years)									
≤50	48	26(54.2%)	22(45.8%)	0.887	0.020	27(56.3%)	21(43.8%)	0.413	0.671
>50	38	20(52.6%)	18(47.4%)			18(47.4%)	20(52.6%)		
Tumor location									
Left	40	18(45.0%)	22(55.0%)	0.141	2.166	19(47.5%)	21(52.5%)	0.403	0.698
Right	46	28(60.9%)	18(39.1%)			26(56.5%)	20(43.5%)		
Tumor size (cm)									
≤5	36	11(30.6%)	25(69.4%)	<0.001*	13.090	23(63.9%)	13(36.1%)	0.068	3.319
>5	50	35(70.0%)	15(30.0%)			22(44.0%)	28(56.0%)		
Tumor grade (differentiation)									
Well	29	22(75.9%)	7(24.1%)	0.003*	8.804	14(48.3%)	15(51.7%)	0.592	0.288
Moderately or poorly	57	24(42.1%)	33(57.9%)			31(54.4%)	26(45.6%)		
Metastasis									
Yes	24	17(70.8%)	7(29.2%)	0.045*	4.026	19(79.2%)	5(20.8%)	0.002*	9.614
No	62	29(46.8%)	33(53.2%)			26(41.9%)	36(58.1%)		
Venous invasion									
+	16	13(81.3%)	3(18.8%)	0.014*	6.090	13(81.3%)	3(18.7%)	0.010*	6.593
–	70	33(47.1%)	37(52.9%)			32(45.7%)	38(54.3%)		
Satellite lesions									
+	24	13(54.2%)	11(45.8%)	0.937	0.006	17(70.8%)	7(29.2%)	0.033*	4.571
–	62	33(53.2%)	29(46.8%)			28(45.2%)	34(54.8%)		
Tumor number									
Solitary	65	32(49.2%)	33(50.8%)	0.164	1.940	35(53.8%)	30(46.2%)	0.619	0.247
Multiple	21	14(66.7%)	7(33.3%)			10(47.6%)	11(52.4%)		
AJCC TNM stage									
I and II	24	4(16.7%)	20(83.3%)	<0.001*	18.143	13(54.2%)	11(45.8%)	0.832	0.045
III and IV	62	42(67.7%)	20(32.3%)			32(51.6%)	30(48.4%)		
AFP (ng/ml)									
≤400	18	7(38.9%)	11(61.1%)	0.163	1.950	9(50.0%)	9(50.0%)	0.824	0.049
>400	68	39(57.4%)	29(42.6%)			36(52.9%)	32(47.1%)		

* Statistically significant difference.

RETRACTED

### Correlation between Notch1 and Notch3 Expression and Prognosis of HCC Patients

A Kaplan-Meier postoperative survival curve was used to evaluate the overall survival rate of HCC patients in relation to Notch1 and Notch3 expression. The log-rank test showed that the survival time was significantly different between the low and high Notch1 (P<0.001) and Notch3 (P<0.001) expression groups. Moreover, the low Notch1 and Notch3 expression groups had better survival (Fig. 1 i and j). But the survival time between the high Notch1 and Notch3 groups had not different (Fig. S1). The cumulative 5-year survival rates were 30.0% and 26.8% in the low Notch1 and Notch3 expression group, respectively, and only 15.2% and 8.9% in the high Notch1 and Notch3 expression groups, respectively.

For Notch1 expression, a univariate Cox regression analysis showed that tumor size, metastasis, venous invasion, tumor number, AJCC TNM stage, and Notch1 protein expression were significantly associated with overall survival (Table 2). Furthermore, to evaluate the potential of high Notch1 expression as an independent predictor for overall survival of HCC, multivariate Cox regression analyses were performed. Although other characteristics failed to demonstrate an independent prognostic role, tumor size, metastasis, venous invasion, tumor number, and Notch1 expression may play a role in the prediction of overall survival in HCC (Table 2). However, in the data for Notch3 expression, a univariate Cox regression analysis also showed that metastasis, venous invasion, AJCC TNM stage, and Notch3 protein expression were significantly associated with overall survival (Table 3). Multivariate Cox regression analyses showed that metastasis, venous invasion and Notch3 expression may play a role in the prediction of overall survival in HCC (Table 3).

**Table 2:** Univariate and multivariate analysis for overall survival of 86 patients (analyze data of Notch1 expression).

Tumor characteristic	Relative risk (95% CI)	P-value
Univariate		
Gender	0.664(0.407–1.083)	0.101
Age (years)	1.472(0.907–2.388)	0.118
Tumor location	0.852(0.525–1.383)	0.517
Tumor size	2.026(1.210–3.392)	0.007*
Tumor grade (differentiation)	0.712(0.427–1.188)	0.193
Metastasis	25.045(10.773–58.225)	<0.001*
Venous invasion	23.858(10.333–55.088)	<0.001*
Satellite lesions	1.587(0.938–2.684)	0.085
Tumor number	2.266(1.325–3.876)	0.003*
AJCC TNM stage	4.940(2.544–9.593)	<0.001*
AFP (ng/ml)	1.231(0.672–2.258)	0.501
Notch1	2.353(1.434–3.859)	0.001*
Multivariate		
Tumor size	3.296(1.245–8.725)	0.016*
Metastasis	18.415(5.968–56.825)	<0.001*
Venous invasion	7.625(2.631–22.096)	<0.001*
Tumor number	2.790(1.522–5.116)	0.001*
AJCC TNM stage	1.034(0.313–3.418)	0.956
Notch1	1.787(1.012–3.155)	0.045*

95% CI: 95% confidence interval.

* Statistically significant difference.

RETRACTED

**Table 3:** Univariate and multivariate analysis for overall survival of 86 patients (analyze data of Notch3 expression).

Tumor characteristic	Relative risk (95% CI)	P-value
Univariate		
Gender	0.856(0.531–1.379)	0.523
Age (years)	1.062(0.664–1.696)	0.802
Tumor location	0.996(0.624–1.590)	0.988
Tumor size	1.105(0.682–1.789)	0.686
Tumor grade (differentiation)	0.674(0.414–1.100)	0.114
Metastasis	8.965(4.845–16.590)	<0.001*
Venous invasion	18.410(8.600–39.407)	<0.001*
Satellite lesions	1.395(0.830–2.345)	0.209
Tumor number	1.352(0.798–2.289)	0.262
AJCC TNM stage	2.328(1.311–4.136)	0.004*
AFP (ng/ml)	0.925(0.522–1.639)	0.790
Notch3	2.848(1.743–4.654)	<0.001*
Multivariate		
Metastasis	3.142(1.352–7.300)	0.008*
Venous invasion	8.774(3.143–24.492)	<0.001*
AJCC TNM stage	1.787(0.969–3.296)	0.063
Notch3	3.114(1.853–5.233)	<0.001*

95% CI: 95% confidence interval.

* Statistically significant difference.

### siRNA can Efficiently Down-regulate Notch1 and Notch3 Expression

The mRNA and protein expression levels of Notch1 and Notch3 were significantly up-regulated in HCC cells compared with HL7702 cells. In particular, in parallel with the increase in metastatic potential in HCC cells (MHCC97H>SMMC7721>HepG2), the mRNA and protein expression levels of Notch1 and Notch3 were markedly up-regulated (Fig. S2a and S2b). The migration and invasion capacity was lowest in HepG2 cells and highest in MHCC97H cells. Therefore, we only used HepG2 and MHCC97H cells for the subsequent experiments. In HepG2 and MHCC97H cells, siRNA down-regulated the expression of Notch1 and Notch3 mRNA and protein levels (Fig.S2c–f). To further confirm that the inhibitory effects of siRNA on Notch1 and Notch3 expression were independent of apoptosis, we used an MTT assay to detect Notch1 and Notch3 siRNA-transfected cells. As the results of the MTT assay show, Notch1 and Notch3 siRNA had no effect on the cell growth or viability of HCC cells (Fig. S2 g).

RETRACTED

### Notch1 and Notch3 Play Different Roles in the Migration and Invasion of HCC Cells

Using transwell cell culture chambers, we measured the migration and invasion of Notch1 and Notch3 siRNA-transfected HepG2 and MHCC97H cells. HepG2 and MHCC97H cells transfected with control siRNA were used as controls. Only Notch1 down-regulation significantly decreased the numbers of migratory HCC cells (Fig. 2a–c). However, Notch1 or Notch3 down-regulation significantly decreased the numbers of invasive HCC cells (Fig. 2d–f). These data indicated that Notch1 down-regulation can reduce the migration and invasion of HCC cells. However, Notch3 down-regulation had no effect on migration and could only reduce invasion in HCC cells. Furthermore, to determine the potential mechanisms of Notch1 and Notch3 in the migration and invasion of HCC cells, we examined the effect of down-regulated Notch1 and Notch3 on metastasis-associated molecules, such as CD44v6, E-cadherin, MMP-2, MMP-9, and uPA. As Fig. 3a shows, Notch1 down-regulation decreases the protein expression of CD44v6, MMP-2, MMP-9, and uPA while increasing the protein expression of E-cadherin in HCC cells. However, Notch3 down-regulation only decreased the protein expression of MMP-2, MMP-9, and uPA.

**Figure 2:** Down-regulation of Notch1 or Notch3 can decrease the migration and invasion of HepG2 and MHCC97H cells in vitro. (a–c) Migrated HCC cells analyzed by transwell assays compared with siRNA controls. (d–f) Invaded HCC cells analyzed by transwell assays compared with siRNA controls. The data are presented as the mean ± SD, *P<0.05 compared with control siRNA-transfected HepG2 cells; #P<0.05 compared with control siRNA-transfected MHCC97H cells. NT: No transfection; Cs: control siRNA transfection; N1s: Notch1 siRNA transfection; N3s: Notch3 siRNA transfection.

**Figure 3:** Effects of down-regulated Notch1 or Notch3 on the expression of CD44v6, E-cadherin, MMP-2, MMP-9, uPA, COX-2, ERK1/2, and p-ERK1/2 in HepG2 and MHCC97H cells. (a) The protein expression of CD44v6, E-cadherin, MMP-2, MMP-9, and uPA was measured by western blot analysis in differently treated HCC cells. (b) The protein expression of COX-2, ERK1/2 and p-ERK1/2 were measured by western blot analysis in differently treated HCC cells. NT: No transfection; Cs: control siRNA transfection; N1s: Notch1 siRNA transfection; N3s: Notch3 siRNA transfection.

### Notch1 and Notch3 Play Different Roles in Regulating COX-2 and the ERK1/2 Pathway

COX-2 can regulate the expression of CD44v6 and E-cadherin, while the ERK1/2 pathway can regulate the expression of MMP-2, MMP-9, and uPA in some cancers. In HCC cells, inhibitors of COX-2 can also effectively decrease the expression of CD44v6 and increase the expression of E-cadherin (Fig. S3). Inhibitors of ERK1/2 can effectively decrease the expression of MMP-2, MMP-9, and uPA (Fig. S4). But it was unknown that if the regulated roles of COX-2 or ERK1/2 were via regulating Notch1 or Notch3. We also examine the proteins expression of Notch1 or Notch3 in HepG2 and MHCC97H cells treated with inhibitors of COX-2 or ERK1/2. As Fig. S5 and Fig. S6 showed, the inhibitors of COX-2 or ERK1/2 can not affect the expression of Notch1 and Notch3 in protein level. Further, we explored the effect of down-regulated Notch1 or Notch3 on COX-2 and the ERK1/2 pathway. As Fig. 3b shows, down-regulated Notch1 decreased the expression of COX-2 and p-ERK1/2. However, down-regulated Notch3 only decreased the expression of p-ERK1/2.

RETRACTED

## Discussion

The Notch pathway interacts with several other signal transduction pathways, and its activation can lead to different outcomes ranging from the control of proliferation to apoptosis, differentiation, and cell fate decision [2]. The Notch pathway includes Notch ligands, receptors, negative and positive modifiers, and Notch target transcription factors. To date, four Notch receptors (Notch1-4) have been identified in mammals. But different Notch receptors play a paradoxical role, either as a tumor suppressor or oncogene. Notch1 and Notch3 are up-regulated in many types of tumors and are involved in the metastasis of tumor cells [3]–[8], [11]–[17]. It has also been reported that high levels of Notch1 and Notch3 expression are related to poor overall survival rates in cancer [9], [10], [18]–[20].But in many tumor, Notch2 may play the opposite roles. The expression of Notch2 was down-regulated in HCC, colorectal cancer, and breast cancer [8], [21], [22]. Low levels of Notch2 expression are related to poor overall survival rates and poor differentiation in cancer [21], [22]. Though Notch4 levels are up-regulated in tumor and involved in tumor [23], [24], Notch4 appears to have committed vascular functions. Notch4 (as a endothelial arterial markers) are expressed by vascular endothelial cells [25] and are involved in sprouting angiogenesis [26]. So it indicated Notch1 and Notch3 may play similar role in tumor cells. However, the research about Notch1 and Notch3 in HCC is limited, especially, the relationships between Notch1 and Notch3 and the prognosis of HCC patients is unknown.

In the present study, we examined the expression of Notch1 and Notch3 by immunohistochemistry in HCC samples as other researchs [27]–[30]. Though immunohistochemistry is a good tool to detect a specific protein expression, while it is not a good tool for quantify a specific protein expression. Western blotting may be good for quantify a specific protein expression. But Notch1 expression in tumor vasculature and is known to be involved in vascular endothelial cells [25]. If total tissue proteins (perhaps including vascular cells) were subjected to western blotting, tumor vascular endothelial cells, in addition to tumor cells, might be evaluated in western blotting. To confirm the results precisely, figures of immunohistochemistry will give us the definite information on distribution and intensity of Notch1 protein both within tumor itself and within tumor vasculature. By using immunohistochemistry, we showed that in tumor tissues, high levels of Notch1 expressions were correlated with tumor size, tumor grade, metastasis, venous invasion and TNM stage, whereas Notch3 expression was correlated with metastasis, venous invasion and satellite lesions. These clinical parameters are also indications of an advanced tumor. The results strongly suggested that Notch1 and Notch3 may play key roles in the advancement of HCC. Prognostic molecular biomarkers are invaluable for the clinician to evaluate patients and to aid in tumor control. The Kaplan-Meier analysis of the survival curves showed a significantly worse overall survival rate for patients whose tumors had high Notch1 (log-rank test, P<0.001) and Notch3 (log-rank test, P<0.001) levels, indicating that high Notch1 and Notch3 protein levels are markers of poor prognosis for patients with HCC. But overall survival rate between high Notch1 and Notch3 was not statistical different (log-rank test, P>0.005). Moreover, a multivariate analysis showed Notch1 and Notch3 expression to be indicators of worse outcomes independent of the known clinical prognostic indicators. These data suggest that high Notch1 or Notch3 expression was correlated with worse outcomes and might be independent prognostic factors for patients with HCC. Thus, expression of Notch1 or Notch3 could constitute a useful additive prognostic marker to the TNM staging system for patients who are more likely to have disease recurrence and are thus good candidates to receive aggressive adjuvant chemotherapeutic treatment. Our present findings suggest that not only Notch1 but also Notch3 can be good for determining the prognosis of HCC patients. However, there is no consensus on which protein plays the predominant role in HCC, thus limiting their clinical predicative value for the prognosis of HCC patients.

RETRACTED

Metastasis is an important factor that affects the prognosis of HCC patients. Metastasis is responsible for cancer-associated mortality, yet it remains the most poorly understood component of cancer. For individual and small groups of cancer cells to break away from the primary tumor and initiate the metastatic process, these cells must acquire the ability to migrate and invade. These traits enable cells to degrade and move through the extracellular matrix of the surrounding tissue toward blood and lymphatic vessels, which in turn provide highways for their passage to distant secondary sites. Thus, to determine which one of Notch1 or Notch3 played the more predominant role in HCC, we focused on evaluating the roles of Notch1 and Notch3 in HCC migration and invasion, which are two important processes of metastasis in vitro.

Adhesion processes are involved at all levels of the migration cascade. Most of the adhesion receptor families reported so far, including integrins, cadherins, selectins, immunoglobulins, and proteoglycans, play a significant role in various stages of tumor progression and metastasis. In our experiments, we focused on two important adhesion molecules, CD44v6 and E-cadherin. The CD44 family comprises important cell adhesion molecules. One of its variants, CD44v6, regulates tumor progression and metastasis formation [31]. Previous reports have indicated that the over-expression of CD44v6 is correlated with the poor prognosis of human cancers [32], [33]. E-cadherin, a member of the cadherin family, is involved in homotypic, calcium-dependent cell-cell adhesion in epithelial tissues [34]. A great deal of previous research has shown that a reduction in E-cadherin is relevant for tumor migration, metastasis, and unfavorable prognosis [35], [36], [37]. The loss of E-cadherin expression and disassembly of E-cadherin adhesion plaques on the cell surface enable tumor cells to disengage from the primary mass and move through conduits of dissemination [38]. In the present study, it was interesting that Notch1 down-regulation could reduce the migration of HCC cells, whereas Notch3 down-regulation could not. A potential explanation could be that Notch1 down-regulation can decrease the protein expression of CD44v6 and increase the protein expression of E-cadherin. Conversely, down-regulated Notch3 had no effect on the protein expression of CD44v6 or E-cadherin.

The Notch signaling pathway is required to convert the hypoxic stimulus into changes in E-cadherin, for increased motility, and for the migration of cervical, colon, glioma, and ovarian cancer cells [39]. In contrast, Lim et al. demonstrated that the Notch1 intracellular domain (N1ICD) can increase the expression of E-cadherin, thereby resulting in a decrease in the invasion of Snail-dependent HCC cells [40]. In the present study, we found that down-regulated Notch1 can increase the expression of E-cadherin, which is involved in cancer invasion and migration. Our results are consistent with the results shown by Wang et al. [41]. The mechanism through which Notch1 mediates E-cadherin regulation in tumor cells is complex and depends on the tissue and cell type. In contrast, the relationship between Notch3 and E-cadherin is unknown. Moreover, the relationship between Notch1 or Notch3 and CD44v6 is unclear. To further explore the mechanism by which Notch1 but not Notch3 can regulate the expression of E-cadherin and CD44v6, we focused on one important pathway, COX-2, which is upstream of CD44v6 and E-cadherin [42], [43]. Tumor COX-2 plays important roles in regulating diverse cellular functions under physiologic and pathologic conditions [44], [45]. Elevated COX-2 expression is often associated with metastasis in cancer [42], [46]. COX-2 contributes to the modulation of E-cadherin and CD44v6 expressions which are involved in cancer metastasis [42], [43]. Knowledge about the relationship between the Notch signaling pathway and COX-2 is limited. One previous study showed that Notch1 can regulate COX-2 expression in gastric cancer through N1IC bound to a COX-2 promoter [47]. In contrast, the relationship between Notch3 and COX-2 is unknown. The results of the current experiments show that down-regulated Notch1 can decrease the expression of COX-2, whereas down-regulated Notch3 cannot. On other hand, inhibition of COX-2 can not affect the protein expression of Notch1 and Notch3. Thus, we speculated that the Notch signaling pathway played different roles in regulating the expression of COX-2. We also speculated that Notch3 cannot affect migration in HCC because Notch3 cannot regulate the expression of COX-2. However, many factors are involved in cancer migration. Our results may demonstrate one possible mechanism. If there are other mechanisms, further studies should be conducted. Our findings suggested that during the migration process of HCC cells, Notch1 is more important than Notch3.

RETRACTED

We also examined whether Notch1 or Notch3 is more important in invasion, which is another process in metastasis. Tumor metastasis occurs by a series of steps, including cell invasion, and the degradation of basement membranes and the stromal extracellular matrix, ultimately leading to tumor cell metastasis. Many molecules are involved in tumor invasion, such as matrix metalloproteinases (MMPs) and urokinase-type plasminogen activator (uPA). MMPs are a family of related enzymes that degrade the extracellular matrix (ECM). Additionally, the activation of these enzymes allows tumor cells to access the vasculature, invade target organs, and develop into tumor metastases [48]. Among the previously reported human MMPs, MMP-2 and MMP-9 play the most important role in tumor invasion and metastasis because of their specificity for type IV collagen, which is the principal component of the basement membrane [49], [50]. The plasminogen activator system is involved in multiple physiological and pathologic processes, including cell migration, angiogenesis, wound healing, embryogenesis, tumor growth, and metastasis. uPA binds to its receptor (uPAR), which facilitates the conversion of plasminogen to plasmin. Plasmin, either directly or indirectly through metalloproteinases (MMP), can degrade components of the extracellular matrix, contributing to cancer cell invasion and metastases [51]. In the present study, Notch1 and Notch3 showed no difference in regulating invasion by HCC cells. Not only down-regulated Notch1 but also down-regulated Notch3 can reduce the invasion of HCC cells. The potential mechanism may be that Notch1 and Notch3 can both regulate the expression of MMP-2, MMP-9, and uPA.

ERK1/2 belongs to the family of mitogen-activated protein kinases (MAPKs), which play a major role in signaling pathways concerning scattering/motility, invasion, proliferation and survival [52], [53]. ERK1/2 activation has also been reported to regulate the expression of a variety of important genes in some cellular responses, including metastasis-related genes, such as MMP-2/−9 and uPA [54], [55]. Because the ERK1/2 pathway plays important roles in many cellular processes, studies on the interaction of ERK1/2 activation with other cell signal transduction pathways, including the Notch signaling pathway, have received increased attention in recent years. Our findings suggest that down-regulated Notch1 and Notch3 can decrease the expression p-ERK1/2, whereas ERK1/2 inactivation can decrease the expression of MMP-2/−9 and uPA. On other hand, inhibition of ERK1/2 can not affect the protein expression of Notch1 and Notch3. This may be one mechanism through which Notch1 and Notch3 are involved in invasion by HCC.

During the study, we found another interesting result. Down-regulated Notch1 and Notch3 did not affect the cell growth or viability of HepG2 and MHCC97H cells. However, Li et al. showed that Notch1 down-regulation inhibits tumor growth in the human HCC cell lines HEP3B, SK-Hep-1 and SNU449 [56], whereas Qi et al. showed that Notch1 over-expression was able to inhibit the growth of SMMC7721 cells [57]. These results also indicated that Notch1 plays a complex role in tumor cells and depends on the tissue and cell type. However, a similar role for Notch3 is unknown. Many studies need to be performed. Thus, the Notch signaling pathway plays a critical role in maintaining the balance between cell proliferation and apoptosis. Moderate changes in the Notch signaling pathway may be caused by the cells’ self-regulation mechanisms, which can protect cells and keep them from being damaged. Non-spontaneous changes in the Notch signaling pathway may affect the results of the experiment and is a limitation of our study.

RETRACTED

In summary, our findings strongly suggested that high levels of Notch1 and Notch3 expression were significantly correlated with HCC progression and unfavorable prognosis. Thus, Notch1 and Notch3 expression can be used as an adjunct to the TNM staging system to improve prognostication for individual patients. Further, we can conclude that Notch1 may interact with more signal transduction pathways related to HCC metastasis than Notch3 from the results above. Therefore, based on the migration and invasion of HCC, we hypothesize that targeting Notch1 in specific cell types may be more useful than Notch3. Additionally, in the near future, targeting the Notch pathway may be used for devising novel preventive and therapeutic strategies for HCC. Furthermore, more mechanisms of Notch1 and Notch3 involvement in HCC should be explored.

## Supporting Information

Figure S1 **Kaplan-Meier statistical analyses of postoperative survival curves according to Notch1 and Notch3 high expression.**
(TIF)

Figure S2 **siRNA can effectively inhibit the expression of Notch1 and Notch3 mRNA and protein levels in HCC cells.** (a and b) RT-PCR and western blot analysis of the mRNA and protein expression level of Notch1 and Notch3 in different HCC cells. (c–f) RT-PCR and western blot analysis of the mRNA and protein expression of Notch1 and Notch3 in differently treated HepG2 and MHCC97H cells. (g) MTT analysis of the cell viability of differently treated HepG2 and MHCC97H cells. The expression of Notch1 and Notch3 was normalized to GAPDH (Notch1 or Notch3/GAPDH). The data are presented as the mean ± SD, *P<0.05 compared with control siRNA-transfected HepG2 cells; #P<0.05 compared with control siRNA-transfected MHCC97H cells. NT: No transfection; Cs: control siRNA transfection; N1s: Notch1 siRNA transfection; N3s: Notch3 siRNA transfection.
(TIF)

Figure S3 **Effects of COX-2 inhibitors on the protein expression of CD44v6 and E-cadherin in HepG2 and MHCC97H cells.** The protein expression of CD44v6 and E-cadherin was measured by western blot analysis. The HepG2 and MHCC97H cells were treated with 50 µmol/l NS-398 and 70 nmol/l SC58125 for 48 h. Cells were treated with DMSO as a control.
(TIF)

Figure S4 **Effects of ERK1/2 pathway inhibitors on protein expression of MMP-2, MMP-9 and uPA in HepG2 and MHCC97H cells.** Protein expressions of MMP-2, MMP-9 and uPA were measured by western blot analysis. The HepG2 and MHCC97H cells were treated with 10 µmol/l PD98059 and 1 µmol/l U0126 for 48 h. Cells were treated with DMSO as a control.
(TIF)

Figure S5 **Effects of COX-2 inhibitors on the protein expression of Notch1 and Notch3 in HepG2 and MHCC97H cells.** The protein expression of Notch1 and Notch3 was measured by western blot analysis. The HepG2 and MHCC97H cells were treated with 50 µmol/l NS-398 and 70 nmol/l SC58125 for 48 h. Cells were treated with DMSO as a control.
(TIF)

Figure S6 **Effects of ERK1/2 pathway inhibitors on protein expression of Notch1 and Notch3 in HepG2 and MHCC97H cells.** Protein expressions of Notch1 and Notch3 were measured by western blot analysis. The HepG2 and MHCC97H cells were treated with 10 µmol/l PD98059 and 1 µmol/l U0126 for 48 h. Cells were treated with DMSO as a control.
(TIF)
